RETRACTED

# Clinical Efficacy and Psychological Impact of Omaha-Based Continuing Care for Prostate Cancer Patients

**DOI:** 10.1155/2022/8735363

**Published:** 2022-07-05

**Authors:** Lanfang Luo, Fangfang Wang, Ling Wang, Jing Zhang, Xiaoyu Liu, Weifen Wang

**Affiliations:** ^1^Urology Surgery, Wuhan No.1 Hospital, 43000, China; ^2^Urology Surgery, Wuhan Third Hospital Tongren Hospital of Wuhan University, 43000, China; ^3^Taizhou Vocational & Technical College, 31800, China; ^4^Emergency Department, Taizhou First People's Hospital, 31800, China

## Abstract

Prostate cancer is a common malignancy elderly male urogenital system, because of the special disease position, and postoperative complications such as urinary retention, urinary incontinence, and sexual dysfunction, if not treated, can increase the patients' physical pain, anxiety, and other psychological burden; endocrine therapy after surgery can affect self-image and quality of life of patients. Omaha system was originally used for community health nurses, which contains three main contents: problem classification, nursing intervention, and outcome evaluation. The problem classification dimension includes four dimensions: environment, physiology, social psychology, and health-related behavior. The nursing intervention dimension is composed of 75 intervention objectives and four behavior types. Omaha system is a nursing intervention model based on individual psychological, physiological, educational level, and family and social background. The model has good clinical application effect. This study aimed to explore the continuous nursing intervention effect in the nursing of patients with prostate cancer and its psychological impact. A total of 96 prostate patients with cancer who were admitted to Taizhou First People's Hospital from November 2019 to May 2021 were divided into Omaha system care group and routine care group with 48 cases each by random number table method. The routine care group received routine care and discharge guidance, and the Omaha system care group on the basis of the routine care group; continuation care based on the Omaha system was implemented. The differences in mental state, life quality score, serum prostate specific antigen (PSA) level, average urine flow rate, and self-care ability score were compared between the routine care and Omaha system care group. The results showed that Omaha-based continuation care for prostate cancer is beneficial to reduce bad mood, improve patients' life quality score and self-care ability, and provide certain reference for clinical care of prostate cancer patients.

## 1. Introduction

Omaha system is an example of standardized terms, the first in the early 1970s by the Visiting Nurse Association of Omaha (VNA) practitioners developed as a home visit service document management system; its theoretical basis is the problem solving method proposed by Weed, which consists of three basic steps: problem, intervention, and outcome. The first step is the Problem Classification Scheme (PCS), in which healthcare practitioners collect information and data to identify patients' nursing problems. The system includes four fields of environment, physiology, social psychology, and health-related behavior, with a total of 42 nursing problems. Each care problem corresponds to different signs and symptoms and is modified with two sets of modifiers (personal, family or community, existing, potential, or health promotor-related). The second step, the Intervention Scheme (IS), contains four types of intervention: health education, guidance and consultation, treatment and procedure, and case management and supervision. There are altogether 75 specific intervention directions, and each intervention category and direction has a standardized definition for standardizing the nursing Intervention process. The last step is the Problem Rating Scale for Outcomes (PRSO), which uses the Likert-type scale structure to evaluate outcomes and intervention effects of each problem from three aspects of cognition, behavior, and state. The evaluation time point can be set and adjusted according to the type and characteristics of the disease. Due to the Omaha system's high efficiency in guiding clinical nursing practice and classifying and integrating nursing information, Not only is it included in the National Library of Medicine's Unified Medical Language System (UMLS) generic index table, logical observation identifiers, names and codes, and systematic Nomenclature of Medicine -- Clinical Terms (SNOMED CT). It is also widely used in community electronic health record system and plays an increasingly important role in the establishment of community residents' health records and the realization of population health assessment data information transmission and exchange. In addition, the Omaha system enables healthcare professionals to understand patients' healthcare needs, enabling clinical data to be valuable in improving and supporting patient-centered clinical practice, education, and research. Today, the Omaha system is more and more widely used in different educational, research institutions and practices abroad.

RETRACTED

Prostate cancer is a common malignancy of the genitourinary system in elderly men, and the current treatment is mainly surgical treatment, of which laparoscopic radical resection of prostate cancer has become the gold standard for surgical treatment [1]. Due to the particularity of the disease site, and postoperative complications such as urinary retention, urinary incontinence, and sexual dysfunction, if not treated in time, it will increase the patient's psychological burden such as physical pain and anxiety, and postoperative endocrine therapy will affect the patient Self-image and life quality [2]. Therefore, giving correct health guidance to patients discharged from radical prostate cancer surgery is of great significance in improving the ability of patients and their families to manage the disease [3]. The Omaha system is a nursing intervention model based on many factors such as individual patients' psychology, physiology, education level, and family and social background. The model has a good clinical application effect [4]. Studies have found that the Omaha system has a good effect in patients with hypertension, lung diseases, and urostomy, but it is less used in patients undergoing radical prostatectomy [5]. Continuing care refers to the ability of patients to continue to receive professional medical care after leaving the original medical environment to promote health recovery [6]. Chronic continuation care is the continuation of hospital care so that patients can obtain comprehensive and continuous nursing services after they are discharged from the hospital and meet the various nursing needs of patients [7]. The Omaha system is a nursing intervention model based on many factors such as individual patient's psychology, physiology, education level, and family and social background. This model has a good clinical application effect [8]. Based on this, this study explores the effect of continuous nursing intervention in the nursing of prostate cancer patients and its impact on patients' psychology. The current research report is as follows.

## 2. Materials and Methods

### 2.1. Research Object

Select 96 patients with prostate cancer admitted to Taizhou First People's Hospital from November 2019 to May 2021, and enroll the patients first to number 96, and then place all the numbers in a closed container, and randomize each patient admitted from the container. Draw 1 number, and put the patient into the corresponding group until both groups of research objects are collected. Before the start of the study, consult with the head of the department, the head nurse, and the prostate cancer specialist, and divide the patients in the Omaha system care group and the routine care group into different wards until the end of the study. Then, the 96 patients were randomly divided into Omaha system care group (48 cases) and routine care group (48 cases) by a random number table method. The Omaha system care group was 52-76 (68.13 ± 4.77) years old, which is composed as follows: (1) junior high school and below: 8 cases; (2) high school and technical secondary school: 22 cases; and (3) junior college and above: 18 cases. 28 cases of adenocarcinoma, 20 cases of squamous cell carcinoma; main caregivers: There are 38 spouses and 10 children. The age of the routine care group was 51~75 (677.66 ± 4.51) years. Education level was as follows: (1) junior high school and below: 20 cases; (2) high school and technical secondary school: 20 cases; and (3) junior college and above: 8 cases. 26 cases of adenocarcinoma, 22 cases of squamous cell carcinoma; main caregivers: There were 37 spouses and 11 children. General information between the routine care and Omaha system care group has no difference (*P* > 0.05).

RETRACTED

### 2.2. Inclusion and Exclusion Criteria

Inclusion criteria is as follows: (1) The included patients meet the “Chinese Expert Consensus on Chemotherapy for Metastatic Prostate Cancer (2019 Edition)” [9]. Diagnostic criteria for prostate cancer, primary school education or above, clear consciousness, no mental or language barriers, and able to communicate well; (2) Basically take care of themselves, use the telephone, primary school education or above, and have complete language skills, There is at least one caregiver at home who can use WeChat and other communication equipment; (3) Patients are willing to participate in the study and are willing to undergo regular follow-up, and patients and family members have signed informed consent forms. Exclusion criteria: (1) Patients with other severe acute and chronic diseases and mental illnesses who are participating in other interventional studies or who have participated in related studies in the past six months; (2) Patients with low expected 1-year survival rate and poor prognosis, prostate The cancer is the metastasis of other malignant tumors rather than the primary cancer; (3) Those who have mental consciousness disorder, have decreased understanding and judgment, do not understand this research, and refuse to participate in this research.

### 2.3. Intervention Methods

The routine care group used routine nursing and discharge guidance, that is, giving perioperative routine nursing and discharge guidance, including the establishment of personal files, distribution of health education manuals (including diet, exercise, medication, psychology, complication monitoring, and follow-up), rehabilitation guidance, and regular follow-ups (including telephone, outpatient, and home follow-up), and requiring patients to write a self-management log.

On the basis of the routine care group, the Omaha system care group implemented Omaha-based continuity care, namely, (1) health guidance and consultation: collect patient clinical data, conduct one-to-one health education for patients, improve their self-care ability, and assist patients in formulating self-care plans. Give more care and encouragement to help patients solve problems in the nursing process in a timely manner, and enhance patients' confidence in overcoming the disease; push disease-related knowledge and nursing knowledge through various channels such as WeChat, QQ, and public accounts to meet patient consultation needs and guidance in a timely manner. It does a good job in daily care and prevention of complications. (2) Operation process: In the nursing process, nursing staff should fully integrate their own professional knowledge, starting from the patient's condition, and comprehensively assess the patient's physical, mental, health, environment, etc., so that the patient can fully understand their own condition and enhance the degree of cooperation; analyze the patient's discharge After the main nursing needs and existing nursing problems, we should formulate effective improvement measures in time, and solve the nursing problems of patients during the home period through outpatient follow-up visits and WeChat platform, so as to improve the nursing behavior of patients. (3) Case management: formulate personalized nursing plans, start from health education, psychological intervention and other aspects, change patient cognition, enhance patient participation, give full play to their subjective initiative, and maximize the role of various medical resources; Continuous follow-up of patients' nursing problems, timely health education and personalized guidance; comprehensive assessment of patients' conditions, effective solutions to patients' nursing problems, and relevant nursing technical guidance. (4) Last is monitoring: Postoperative monitoring is an important part of continuous nursing intervention. It can check the patient's condition in time, track the situation after discharge, and ensure the effective implementation of various nursing measures; after the patient is discharged, the nursing intervention can be strengthened through WeChat, family visits, telephone follow-ups, etc., Supervise patients to complete relevant nursing content in a timely manner; Wechat follow-up to patients once a week after discharge, carefully inquire about the specific situation of patients after discharge and give targeted guidance, and guide outpatient follow-up visits if necessary. Both care for 3 months continuously.

RETRACTED

### 2.4. Observation Indicators

#### 2.4.1. Serum PSA Level

Serum PSA level was detected after fasting blood sampling.

#### 2.4.2. Urine Flow Rate

Urine flow rate refers to the volume of urine discharged from the body through the urethra per unit time, calculated in ml/s. Urine flow rate is the simplest, non-invasive and non-invasive method in urodynamic examination, which objectively reflects the urination process of the lower urinary tract. It reflects the function of bladder, bladder neck, urethra, and urethral sphincter during voiding and the relationship between them.

#### 2.4.3. Psychological State

The patient's anxiety level is evaluated by the Self-Rating Anxiety Scale (SAS), with a full score of 100; the higher the score, the more severe the patient's anxiety; the patient's depression level is evaluated by the Self-Rating Depression Scale (SDS), with a full score 100; the higher the score, the more severe the patient's depression [4]. Both groups were evaluated at the time of discharge and 3 months after discharge. The Cronbach's *α* values measured before use were all greater than 0.914.

#### 2.4.4. Quality of Life

The patient will be followed up by telephone after 3 months of treatment, and the quality of life will be evaluated: The core scale for cancer patients is used for evaluation. There are 30 items in total. Reference 10 and reference 11 are divided into 7 levels. According to the patient's answer options, from 1 to 7 points; other items are divided into 4 levels: from nothing to a little, more to 4 points, 1 to 4 points directly, usually divided into several aspects. There are 15 domains, divided into 4 functional domains such as physical, cognitive, emotional, and social functions; 3 symptom domains such as fatigue, pain, nausea, and vomiting; 1 overall health status/life quality domain, and 6 individual domains (each as a domain); add the scores of the items contained in each domain, and divide by the number of items contained in the domain to get the score of the domain. Significance of the scoring rules: The more the score for function and overall health, the better the function and the life quality. The higher the score for symptoms, the more symptoms of discomfort and the worse the life quality. The Cronbach's *α* values measured before use were all greater than 0.914. Patients or their accompanying family members should fill out the test independently before treatment and 3 months after treatment without being affected by any internal or external factors. The test will be completed in 57 minutes.

#### 2.4.5. Unhealthy Emotions

Compare the self-care ability scores of the routine care and Omaha system care group of patients, and use the self-care ability measurement scale to evaluate before the intervention and 3 months after the intervention, including 4 items of self-care skills, health knowledge, and self-concept and self-responsibility. There are 43 items, each item scores 0-4 points, and the total score is 172 points. The higher the score, the stronger the patient's self-care ability.

RETRACTED

### 2.5. Statistical Methods

The statistical processing software is SPSS25.0, and the measurement data expressed as mean ± standard deviation ($\bar{x}\pm \text{S}$) using *t* test. Use the Fisher exact probability test or*χ*2test to express the count data in percentage (%); statistically,*P* < 0.05is meaningful.

## 3. Results

### 3.1. Mental States

At the time of discharge, there was no significant difference in SAS and SDS scores between the routine care and Omaha system care group of patients (*P* > 0.05). The SAS and SDS scores of the routine care and Omaha system care group were lower than those at discharge 3 months after discharge, and the SAS and SDS scores of the Omaha system care group 3 months after discharge All were lower than routine care group (P <0.05). See Table 1.

### 3.2. Quality of Life Scores

The life quality scores in the Omaha system care group, such as emotion, cognition, society, and overall health, were significantly higher than those of the routine care group, while the physical, fatigue, nausea, vomiting, and pain were lower than those of the routine care group, which was statistically significant (*P* < 0.05) (see Tables 2 and 3).

### 3.3. Serum PSA Level and Average Urine Flow Rate

The serum PSA level and average urine flow rate of patients in the Omaha system care group were better than those in the routine care group at 3 months after discharge (*P* < 0.05) (Table 4).

### 3.4. Comparison of Self-Care Ability Scores

There was no statistically significant difference in the self-care ability scores of the routine care and Omaha system care group of patients at discharge (*P* > 0.05). The self-care skills score, self-responsibility score, health knowledge score, and self-concept score of the Omaha system care group were better than the control at 3 months after discharge (*P* < 0.05) (details in Table 5).

## 4. Discussion

Radical prostatectomy is the most effective and commonly used treatment for prostate cancer, but patients usually have serious psychological problems after surgery, and the body is traumatized, and the patient's postoperative immune status is poor [12–15]. Patients still need professional health guidance after they are discharged. However, routine post-discharge care cannot meet the purpose of comprehensive care for patients [16, 17]. The Omaha system was first proposed in the United States in the 1970s. This model emphasizes the classification of existing health problems, taking into account the patient's physical, mental, and family background and then establishing comprehensive individualized care to meet the patient's health recovery needs [18–21]. As a more scientific nursing model, continual nursing can further extend hospital care to outside the hospital to ensure that patients can also obtain nursing services and nursing guidance from nursing staff after they are discharged from the hospital so that they can understand their own diseases and actively cooperate with medical staff in their work. Strictly follow the doctor's advice to complete the content of home self-care [22–24]. The continuous care model has been widely used in patients with various clinical diseases [25]. The Omaha system is currently recognized as a nursing system with good results. It is widely used in clinical and community continuity nursing work and can effectively promote the improvement of nursing quality [26]. The Omaha system can comprehensively evaluate the data of the patient and, on this basis, formulate an individualized plan that meets the needs of the patient, better meet the needs of the patient, and promote the patient to recover as soon as possible [27, 28]. Continuous care can provide patients with continuous and high-quality nursing services. If combined with the Omaha system, the advantages of both can be fully utilized to further strengthen the clinical care effect and allow patients to obtain high-quality nursing services during their stay at home [10, 29, 30].

RETRACTED

In this study, it was found that life quality scores of the Omaha system care group were significantly higher than those of the routine care group, such as emotion, cognition, society, and overall health, while the physical, fatigue, nausea, vomiting, and pain were significantly lower than routine care group. The serum PSA level and average urine flow rate of patients in the Omaha system care group were better than those in the routine care group 3 months after discharge. There is no significant difference in the self-care ability scores of the routine care and Omaha system care group at discharge. The scores of self-care skills, self-responsibility scores, health knowledge scores, and self-concept scores of patients in the Omaha system care group after discharge for 3 months were better than routine care group. It shows that Omaha-based continuation care for prostate cancer is beneficial to reduce bad mood and improve the patient's life quality score and self-care ability. In this study, it was found that the SAS scores and SDS scores of patients in the Omaha system care group were lower than those in the routine care group after discharge from the hospital at 3 months. The data suggests that continuation of care based on the Omaha system is beneficial to reduce the patients' adverse mood scores. Analysis of the reason may be due to the emphasis on psychological intervention in the process of early rehabilitation and the explanation of postpartum precautions in the process of psychological intervention, which improves the correct understanding of prostate cancer and postpartum [11, 31]. This study shows that Omaha system application in patients' postoperative continuation care plays an important role in improving self-care ability, helps patients treat their own conditions correctly, and enhances patients' sense of self-efficacy. Analyze the reason: Omaha system model nursing can increase patients' understanding of disease-related knowledge, correct misunderstandings in time, help patients master professional nursing knowledge, improve self-care ability, and ensure the smooth implementation of various nursing tasks [32–34]. At the same time, it alleviates patients' worries, enhances patients' confidence in overcoming the disease, enables patients to maintain a positive attitude towards their own diseases, and obtains ideal care effects [35].

RETRACTED

This study not only provides a reliable nursing experience for patients with radical prostatectomy but also promotes the quality of department care to a certain extent. At the same time, limitations in the number of cases have led to some deficiencies in this study. Factors such as age and education level vary, and the majority of patients are rural elderly patients resulting in insufficient knowledge and awareness of the disease. Therefore, there are relatively few samples in this study; another shortcoming of this study is the short intervention time, and nursing measures continuity needs improvement in the future. In the future, it is necessary to expand the sample size, strengthen the network platform promotion, and extend the intervention time. In summary, the Omaha-based continuation care for prostate cancer is beneficial in reducing bad mood, improving patients' life quality scores and self-care ability, and provides a certain reference for clinical care of prostate cancer patients.

## Figures and Tables

**Table 1:** Mental status scores between the routine care and Omaha system care group ($\bar{x}\pm \text{s}$).

Group	SAS scores	SDS scores
On discharge		
Omaha system care group (*n* = 48)	56.39 ± 4.75	62.23 ± 5.08
Routine care group (*n* = 48)	56.42 ± 4.79	62.25 ± 5.07
*t*	-0.031	0.019
*P*	0.975	0.985
Months discharged		
Omaha system care group (*n* = 48)	32.64 ± 3.31^a^	34.49 ± 3.74^a^
Routine care group (*n* = 48)	45.68 ± 3.47^a^	48.89 ± 3.66^a^
*t*	−18.839	−19.065
*P*	<0.001	<0.001

Note: Compared with on discharge ^a^*P* < 0.05.

RETRACTED

**Table 2:** Quality of life (mental) of the routine care and Omaha system care group of patients ($\bar{x}\pm \text{s}$).

Group	Body	Cognition	Emotion	Society
Routine care group (48)	77.27 ± 10.14	59.27 ± 16.23	62.21 ± 10.21	50.14 ± 10.16
Omaha system care group (48)	70.23 ± 11.57	66.25 ± 16.82	70.23 ± 10.57	55.15 ± 12.45
*t*	3.170	−2.069	−3.781	−2.160
*P*	0.002	0.041	<0.001	0.033

**Table 3:** Quality of life (symptoms) of the routine care and Omaha system care group of patients ($\bar{x}\pm \text{s}$).

Group	Overall health	Feel sick and vomit	Tired	Pain
Routine care group (48)	50.27 ± 10.14	52.27 ± 8.23	54.18 ± 11.68	42.14 ± 5.21
Omaha system care group (48)	59.23 ± 10.57	48.25 ± 8.82	46.23 ± 10.57	34.15 ± 5.64
*t*	−4.238	2.819	3.496	7.210
*P*	0.001	0.006	0.001	<0.001

**Table 4:** Serum PSA levels and average urine flow rate between the routine care and Omaha system care group ($\bar{x}\pm \text{s}$).

Group	PSA (*μ*g/L)	Mean urine flow rate (ml/s)
On discharge		
Omaha system care group (*n* = 48)	48.39 ± 6.75	1.73 ± 0.48
Routine care group (*n* = 48)	47.42 ± 7.79	1.75 ± 0.27
*t*	0.652	0.252
*P*	0.516	0.802
Months discharged		
Omaha system care group (*n* = 48)	13.64 ± 3.31^a^	64.49 ± 13.74^a^
Routine care group (*n* = 48)	25.68 ± 6.47^a^	54.89 ± 9.66^a^
*t*	−11.478	3.960
*P*	<0.001	<0.001

Note: Compared with on discharge ^a^*P* < 0.05.

**Table 5:** Self-care ability scores of the routine care and Omaha system care group of patients ($\bar{x}\pm \text{s}$).

Group	Self-care skills	Self-responsibility	Health knowledge	Self-concept
On discharge				
Omaha system care group (*n* = 48)	33.56 ± 5.18	17.97 ± 4.43	40.87 ± 8.71	19.58 ± 5.44
Routine care group (*n* = 48)	33.58 ± 4.21	18.95 ± 3.42	41.92 ± 7.73	18.61 ± 4.42
*t*	−0.021	−1.213	−0.625	0.939
*P*	0.983	0.228	0.543	0.350
Months discharged				
Omaha system care group (*n* = 48)	46.79 ± 6.82^a^	29.29 ± 6.06^a^	27.17 ± 8.43^a^	28.94 ± 7.02^a^
Routine care group (*n* = 48)	38.12 ± 8.43^a^	21.87 ± 5.12^a^	21.16 ± 7.42^a^	23.21 ± 6.96^a^
*t*	5.540	6.480	3.708	4.016
*P*	<0.001	<0.001	<0.001	<0.001

Note: Compared with on discharge. ^a^*P* < 0.05.

## Data Availability

No data were used to support this study.
